# APU-Net: An Attention Mechanism Parallel U-Net for Lung Tumor Segmentation

**DOI:** 10.1155/2022/5303651

**Published:** 2022-05-09

**Authors:** Tao Zhou, YaLi Dong, HuiLing Lu, XiaoMin Zheng, Shi Qiu, SenBao Hou

**Affiliations:** ^1^School of Computer Science and Engineering, North Minzu University, Yinchuan, Ningxia 750021, China; ^2^The Key Laboratory of Images and Graphics Intelligent Processing of State Ethnic Affairs Commission, North Minzu University, Yinchuan 750021, China; ^3^School of Science, Ningxia Medical University, Yinchuan, Ningxia 750004, China; ^4^Research Institute for Reproductive Medicine and Genetic Diseases, Wuxi Maternity and Child Health Hospital, Jiangsu Wuxi, 214002, China; ^5^Key Laboratory of Spectral Imaging Technology CAS, Xi'an Institute of Optics and Precision Mechanics, Chinese Academy of Sciences, Xi'an, Shanxi 710119, China

## Abstract

Lung cancer is one of the malignant tumors with high morbidity and mortality, and lung nodules are the early stages of lung cancer. The symptoms of pulmonary nodules are not obvious in the clinic, and the optimal treatment time is missed due to the missed diagnosis in the clinic. A parallel U-Net network called APU-Net is proposed. Firstly, two parallel U-Net networks are used to extract the features of different modalities. Among them, the subnetwork UNet_B extracts the CT image features, and the subnetwork UNet_A consists of two encoders to extract the PET/CT and PET image features. Secondly, multimodal feature extraction blocks are used to extract features for PET/CT and PET images in UNet_B network. Thirdly, a hybrid attention mechanism is added to the encoding paths of the UNet_A and UNet_B. Finally, a multiscale feature aggregation block is used for extracting feature maps of different scales of decoding path. On the lung tumor ^18^FDGPET/CT multimodal medical images dataset, experiments' results show that the DSC, Recall, VOE, and RVD coefficients of APU-Net are 96.86%, 97.53%, 3.18%, and 3.29%, respectively. APU-Net can improve the segmentation accuracy of the adhesion between the lesion of complex shape and the normal tissue. This has positive significance for computer-aided diagnosis.

## 1. Introduction

Lung cancer has become one of the most common cancers, and it is a cancer with the highest fatality rate at present. When lung cancer patients are diagnosed, 70% patients has been already in the middle or advanced stage [1], the five-year survival rate for lung cancer patients is often less than 15% [2]. Hence, there are great significance for the early intervention and treatment of lung cancer patients. In the early stage, the main form of lung cancer is pulmonary nodules. When checked with Computed Tomography (CT), its imaging manifestations are mainly circular shadows with a diameter of no more than 30 mm [3]. With the improvement of medical image imaging technology, the scale of medical imaging data has been increased rapidly, which brings great challenges to the clinical work, and the workload of clinicians is greatly increased by judgment of large amount of medical imaging data. Due to the small area of pulmonary nodules in the whole medical image and the low contrast between the lesion and the background, it is easy to miss a diagnosis. Therefore, the computer-aided diagnosis system for automatic segmentation of pulmonary nodules [4–6] has become a research hotspot. There are outstanding achievements of deep learning methods in the field of image semantic segmentation, such as FCNs [7] and DeepLabV3 [8]. Hence, it can be widely used in medical image segmentation, of which the typical model is U-Net [9]. U-Net is an encoder and decoder structure, which can achieve semantic segmentation of the input images [10] and realize a good segmentation effect in small medical image datasets. Aiming at the problem that the segmentation performance of lung CT images is not high, Khanna et al. [11] added residual blocks to the U-Net network to improve the segmentation performance. Liu et al. [12] input two CT images of different scales into a residual blocks based on dual-path network, and the network encoder extracts the global and local features of the image from residual blocks and rich contextual information of pulmonary nodules. Aiming at the problem of the loss of spatial information caused by U-Net pooling operation, Gridach [13] proposed a pyramid expansion network, which integrates multiple dilated convolutions with different dilated rates to capture the tiny details of the image. Channel attention mechanism is added to skip connection of U-Net for lung parenchymal segmentation by Wang et al. [14], and the last layer of the network used a hybrid dilated attention convolution layer. Some researchers make full use of the target slices and its continuous slices to provide sequence information of lesions and improving the segmentation accuracy. Cao et al. [15] proposed a dual-path residual network for the 3D segmentation of pulmonary nodules. The target slice and two adjacent slices are input into an encoder with an improved residual structure, and a weighted sampling strategy is used for unbalanced training labels. Lee et al. [16] proposed the Mu-net network to be used for 3D image denoising, the downsampling is used to generate images of different scales in the input image, and different scales' images are input different scales' U-Net to extract image features of different scales. However, most of the current segmentation methods only use single-modal medical images, which ignores the complementarity of multimodal medical images to lesions. Therefore, in this paper, a parallel U-Net network is proposed for the lung lesion segmentation in combination with the different abilities of multimodal medical images to characterize lesions and uses a hybrid attention mechanism in this paper.

## 2. Methods

In this study, the paper proposed an attention mechanism parallel U-Net. It could be used for doctors to segment lung lesions and reduce missed diagnoses.

### 2.1. Dataset and Preprocessing

A total of 90 clinical patients with lung tumors are collected, confirmed by surgical pathology, including 32 females and 58 males, between January 2018 and June 2019 at the nuclear medicine department of a hospital in Ningxia. The patients ranged in age from 20 to 87 years, with a mean age of 61.2 ± 13.6 years, the patient's blood glucose is controlled to normal, patients are forbidden to eat for 6 hours and are injected with ^18^F-FDG (^18^F-Nuorodeoxyglucose) 0.11~0.13mci/kg (^18^F-FDG is automatically synthesized by the HM-10 accelerator of Sumitomo, Japan, with a radiochemical purity greater than 95%), and the imaging is performed after approximately 60 minutes of lying down. Before imaging, drink 500 ml of water. To ensure the lesions are annotated correctly, the ground truth is annotated by radiologists with 30 years of experience. After data augmentation processing, such as rotation and mirror image, the final sample number of the three modal image datasets is 1026, respectively, including 909 PET/CT, CT, and PET images as the training set, and 117 PET/CT, CT, and PET images as the testing set. The image labels are manually drawn by clinicians.  Figure 1 shows the contrast between PET/CT and CT images.

To solve the problem that pulmonary nodules occupy too few pixels of the whole image in the original image, ROI extraction based on Hough transform [17] is used to cut the original image to a pixel size of 50 × 50. And an image enhancement method based on exposure fusion [18] is used to improve the contrast between pulmonary nodules and background. The cross-entropy loss function is used for both subnetworks. Adam optimizer is used, training time is 150, the learning rate is initialized to 0.005, and batch size is 8. To prevent network overfitting, dropout is added to the network layer.

### 2.2. APU-Net

Two parallel U-Net (UNet_A and UNet_B) networks are used to extract multimodal medical image features of PET/CT (Positron Emission Tomography/Computed Tomography), CT (Computed Tomography), and PET (Positron Emission Tomography). UNet_A is composed of two encoders (encoder1_A and encoder2_A), which extracts medical image features of PET/CT and PET. UNet_B network extracts the features of CT images. Master network, which is composed of UNet_B, provides rich anatomical structure information for lesion segmentation. These features, that are extracted from the two subnetwork encoder paths, are concatenated and input into the decoder paths through the hybrid attention mechanism. Hence, a mutual image fusion method is realized about multimodal medical image features, to take full advantage of the complementarity of multimodal medical images. PET/CT and PET images are input into the UNet_A encoders, as shown in Figure 2. CT images are input into the UNet_B encoder, as shown in Figure 2. A hybrid attention mechanism is proposed in the skip connection of the network. Input features of UNet_A and UNet_B encoder paths are processed by the attention mechanism and input into decoder_A and decoder_B, respectively. Multiscale feature maps of two decoder paths are aggregated by multiscale feature aggregation blocks, and segmentation results are better than others.

The UNet_A consists of two encoders and one decoder. The UNet_A structure is shown in Figure 3. PET images and PET/CT images are input Encoder1_A and encoder2_A, respectively. The two encoders have the same parameters, and there are five layers. Each encoder layer of UNet_A includes two convolutional blocks, which consist of 3 × 3 convolutional blocks, Batch Normalization (BN), and ReLU activation function. To reduce the parameters of parallel U-Net, the number of convolutions at the first layer of the network is 16. With the deepening of the network, the number of convolution kernels at each layer increases by two times. The convolutional kernel number of the encoder1_A and encoder2_A is 16, 32, 64, 128, and 256, respectively. After each convolution layer, the downsampling operation is connected, and the downsampling operation is the 2 × 2 maximal pooling, and the image size is reduced to half comparing with the beforeimage when each downsampling. At the last layer of the UNet_A network, two-modal medical image features of extracting by the two encoders are summed, and the summed feature maps are input into the decoder_A. Decoder_A consists of four layers, and there are two convolution blocks in each layer, the convolution block is same as the encoder1_A. The convolution kernel number is 128 at the first upsampling, and the number of convolution kernels is reduced to half and the image size is doubled at each upsampling. The upsampling operation of the decoder_A is a 2 × 2 transpose convolution. A two-modal medical image feature extraction block is used for each layer of PET feature maps and PET/CT feature maps of the UNet_A encoder. This feature extraction block is used to extract relevant information by an attention gate from the PET image and PET/CT image, and these feature maps are transmitted to the hybrid attention mechanism of skip connection. The input feature maps of skip connection not only contain the feature maps *F*_*hybrid*_*en*_ of the UNet_A encoder but also receive the feature maps *F*_*CT*_*en*_ of UNet_B which makes the underlying features fuse with each other and realize feature reuse. The UNet_A parameters are shown in Table 1.

The UNet_B has five layers, and the numbers of convolutional kernels for encoder are 32, 64, 128, 256, and 512, respectively. Each layer of the network consists of two 3 × 3 convolutional blocks, Batch Normalization (BN), and activation function ReLU. Downsampling uses a 2 × 2 maximal pooling, and the size of the feature maps is halved after downsampling. There are four layers in decoder_B, and convolutional kernel numbers of each layer are 256, 128, 64, and 32, respectively. Hybrid features *F*_*hybrid*_*en*_ and the UNet_B encoder feature maps *F*_*CT*_*en*_ are input into the decoding paths of two subnetworks through the attention mechanism.  Table 2 describes the UNet_B network parameters, and the UNet_B structure is shown in Figure 4.

#### 2.2.1. Two Modal Medical Image Feature Extraction Block

In the UNet_A, the two-modal medical image feature extraction block is used to extract complementary feature maps of PET and PET/CT. This block includes two input feature maps, namely, *χ*_1_^*l*^ and *χ*_2_^*l*^, as shown in Figure 5.First, *χ*_1_^*l*^ and *χ*_2_^*l*^ are concatenated, then 1 × 1 convolution and ReLU are performed on the concatenated feature maps, and then, 1 × 1 convolution and sigmoid functions are performed to compress the weight of the feature maps to between 0 and 1. Finally, the output weights after sigmoid function are multiplied with the concatenated feature maps. The feature maps are inputted into the skip connection after multiplication, and the formula is expressed as equation (1).

(1) $$\begin{array}{c} F_{hybrid\_en}^{l}=\left(\chi_{1}^{l}+\chi_{2}^{l}\right)⊗\sigma \left({Conv}_{3\times 3}\left({Conv}_{1\times 1}\left(\chi_{1}^{l}+\chi_{2}^{l}\right)\right)\right), \end{array}$$

where *χ*_1_^*l*^ represents the layer *l* PET/CT feature maps extracted by UNet_A, *χ*_2_^*l*^ represents layer *l* PET feature maps extracted by UNet_A, *Conv*_1×1_(·) represents 1 × 1 convolution operation and ReLU function, *Conv*_3×3_(·) represents 3 × 3 convolution operation, “*σ*” represents sigmoid function, and *F*_*hybrid*_*en*_^*l*^ represents the two-modality medical image feature representation of the *l* layer *F*_*hybrid*_*en*_^*l*^ extracted by UNet_A.

#### 2.2.2. Hybrid Attention Mechanism

Hybrid attention mechanism [19] includes spatial attention mechanism and channel attention mechanism. The spatial attention mechanism focuses on the lesion in the feature map and suppresses irrelevant information such as the background information. Channel attention can assign larger weight coefficients to important channel feature maps, so it is necessary to process the attention mechanism of the three modal image features of the skip connection.

*(1) Spatial Attention Mechanism*. First, the UNet_A feature maps *F*_*hybrid*_*en*_ and UNet_B feature maps *F*_*CT*_*en*_ are concatenated and perform the maximal pooling and average pooling on the concatenated feature maps, respectively. The average pooling denoise the lung tumor image, and the maximal pooling highlights the lung tumor in the medical image. Then, the two pooled feature maps are concatenated, 3 × 3 convolution operation is performed on the concatenated feature maps, using sigmoid function to compress the feature coefficients range from 0 to 1, and the original feature maps are multiplied by the weight coefficients, as shown in Figure 6.

Specifically as shown in equation (2), where “*σ*” represents the sigmoid function, “+” represents the concatenating the feature maps. *F*_*hybrid*_*en*_^*l*^ is the two modal medical images feature maps of layer 1 extracted by UNet_A, and *F*_*CT*_^*l*^ is the feature maps extracted by UNet_B. The two-modality medical image feature maps *F*_*hybrid*_*en*_^*l*^ and the CT feature maps *F*_*CT*_*en*_^*l*^ are concatenated, named as *χ*^*l*^. “⊕” represents the summed of the channels feature maps, “⊗” represents the multiplication, and *SA*(·) represents the spatial attention mechanism operation.

(2) $$\begin{array}{c} {SA}^{l}\left(F\right)=\chi^{l}⊕\left[\chi^{l}⊗\left(\sigma \left({Conv}_{3\times 3}\left(AvgPool\left(\chi^{l}\right)+MaxPool\left(\chi^{l}\right)\right)\right)\right)\right]. \end{array}$$

*(2) Channel Attention Mechanism*. First, to utilize more feature information, the average pooling and the maximal pooling are used to process the concatenate feature maps *χ*^*l*^ to obtain two 1 × 1 × C weight coefficients. Then, using the MultiLayer Perceptron (MLP) which composed of two fully connected layers and ReLU function to implement nonlinear transformation of features, the neuron numbers are 1/3 of the number of feature maps channel in the first fully connected layer, activation function is the ReLU function, and the neuron numbers are the feature map channels number in the second fully connected layer. Finally, the two results obtained by MLP are summed, and “*α*” weight coefficient is obtained through sigmoid function, and “*α*” weight coefficients and *χ*^*l*^ feature maps are multiplied and obtained the weighted feature maps, named as *R.* Then channel attention feature maps are obtained through sum weighted feature maps *R* and feature maps *χ*^*l*^. These processing are as shown in Figure 7, and the formula is expressed as

(3) $$\begin{array}{c} {CA}^{l}\left(F\right)=\left(\chi^{l}⊗\sigma \left(MLP\left(avgPool\left(\chi^{l}\right)\right)⊕MLP\left(\max Pool\left(\chi^{l}\right)\right)\right)\right)⊕\chi^{l}. \end{array}$$

### 2.3. Multiscale Feature Aggregation Block

The network decoder contains low-level semantic feature information, and this information plays a vital role in lesion segmentation. Due to their different sizes in different scale feature maps, feature maps have different relevance in different scales to the object. Inspired by the reference [20], a multiscale feature aggregation (MFA) block is used to automatically determine the scale-wise weight for each pixel. The MFA block is illustrated in Figure 8. We concatenate each layer feature maps of decoder_A and decoder_B, and then, bilinear interpolation is used to resample the feature maps of different scales to a size of50pixel × 50pixel, and1 × 1convolution operation is used to compress the four scale feature map channels into 16, and the feature maps were denoted as *F*. Avg-pooling and MLP are performed to obtain the channel coefficients, similar to the channel attention mechanism. The formula is expressed as equation (4). Where “*σ*” represent sigmoid function, and “*α*” represent channel coefficient.

(4) $$\begin{array}{c} \alpha =\sigma \left(MLP\left(avgPool\left(F\right)\right)\right). \end{array}$$

After the channel coefficients “*α*” are multiplied by the concatenated feature maps *F*, 3 × 3 convolution operation, ReLU function, 1 × 1 convolution operation, and sigmoid function are performed to obtain the coefficients “*β*”, as shown in

(5) β=σConv1×1ReLUConv3×3F·α.

Finally, the residual connection is used to connect the features. The specific process is shown in

(6) $$\begin{array}{c} F_{MFA}=F\cdot \alpha \cdot \beta +F\cdot \alpha +F. \end{array}$$

## 3. Experimental Results

### 3.1. Implementation and Evaluation Models

All models are based on the PyTorch framework, cross entropy loss is used for training of UNet_A and UNet_B, Adaptive Moment Estimation (Adam) is used to train the model, and the value of the initial parameter is the following: initial learning rate is 0.005, batch size is 8, weight decay is 10^−7^, iteration epochs are 150, and the model is implemented on one NVIDIA Geforce GTX 1080 Ti GPU.

In order to evaluate the network performance, the DSC, Recall, Volumetric Overlap Error (VOE), and Relative Volume Difference (RVD) are used. The specific formula are as follows. In this paper, the positive values of VOE and RVD are taken, the smaller the value of these two variables are the better. In order to be able to unify these four evaluation indicators, the two indicators of VOE and RVD use the method of calculating the absolute value with 1. The calculation methods of VOE and RVD indicators are as follows:

(7) $$\begin{array}{c} DSC=\frac{2\times \left|P\cap G\right|}{\left|P\right|+\left|G\right|}, \end{array}$$

(8) Recall=TPTP+FN,

(9) $$\begin{array}{c} VOE=abs\left(1-\left|\frac{P\cap G}{P\cup G}\right|\right), \end{array}$$

(10) $$\begin{array}{c} RVD=abs\left(\frac{P}{G}-1\right), \end{array}$$

where the correct segmentation of the lesion area is defined as True Positive (TP), the normal tissue area is segmented as the lesion area is defined as False Positive (FP), and the normal area is segmented as True Negative (TN). Segmentation of the focal area into a normal area is defined as False Negative (FN). *P* represents the target pixel predicted by the model, and *G* represents the target pixel in the ground truth.

### 3.2. Performance of the Model

#### 3.2.1. Network Architecture

In experiment 1, the network model is U-Net. 909 CT images are used as the training sets, and 117 CT images are used as the testing set. In experiment 2, the network model is multiencoder U-Net (MEU-Net), this network is based on U-Net. PET, CT, and PET/CT medical images are input into three encoders, respectively. In the last layer of the network, the feature maps of the three encoders are summed, and the parameters of MEU-Net every layer are the same as U-Net, each network layer uses two 3 × 3 convolution blocks, and convolutional kernels' numbers of each layer are 1024, 512, 256, 128, and 64, respectively. In MEU-Net, we sum the feature maps of the three encoding paths and transmit them to the decoding path through the skip connection. 909 PET/CT, CT, and PET images are used as the training sets, and 117 PET/CT, CT, and PET images are used as the testing set. In experiment 3, the network model is a parallel U-Net network (PU-Net), PU-Net is a network in which APU-Net removes the two-module medical image extraction block, hybrid attention mechanism, and multiscale feature aggregation block. The segmentation results of the UNet_A and UNet_B are summed as the final segmentation result of the PU-Net network. 909 PET/CT, CT, and PET images are used as the training set, and 117 PET/CT, CT, and PET images are used as the testing set. PET/CT and PET images are input into the encoder1_A and encoder2_A, respectively, and CT images are input by the encoder_B. The feature maps of encoder_A and encoder_B are concatenated and transmitted to the corresponding decoder_A and decoder_B through skip connection. The segmentation results of the two subnetworks UNet_A and UNet_B are summed as the segmentation result of the PU-Net. The evaluation indexes of segmentation result are shown in Table 3.  Figure 9 is the CT image three-dimensional gray value and Figure 10 is the network segmentation results.

Figure 10 shows the segmentation results of U-Net, MEU-Net, and PU-Net. It can be seen that the lesion segmentation results of PU-Net are more accurate than U-Net and MEU-Net. In the third row of Figure 10, comparing with the ground truth of lesion in CT image, PU-Net is superior to the other two networks in delineating the lung tumor lesion shape. It is proved that the parallel U-Net is effective in improving the performance of multimodal medical images segmentation.

#### 3.2.2. Attention Mechanism Module

Four experiments are conducted to evaluate segmentation performance of attention mechanisms and multiscale feature aggregation blocks on APU-Net. All experiments are based on the PU-Net, and 909 PET/CT, CT, and PET images are used as the training sets, and 117 PET/CT, CT, and PET images are used as the testing set. In experiment 1, the network model is PU-Net. In experiment 2, the network model is PU-Net based on the spatial attention mechanism and named as SAPU-NET. The feature maps *F*_*hybrid*_*en*_ and *F*_*CT*_*en*_ are concatenated and input into the spatial attention mechanism of skip connection. In experiment 3, the network is PU-Net based on the channel attention mechanism and named as CAPU-Net. The feature maps *F*_*hybrid*_*en*_ and *F*_*CT*_*en*_ are concatenated and input to the channel attention mechanism of skip connection. In experiment 4, the parallel U-Net is based on multiscale feature aggregation block and named as MFPU-Net, and the feature maps of the UNet_A and UNet_B decoder are concatenated and input into the multiscale feature aggregation block. The evaluation indexes of segmentation result are shown in Table 4.  Figure 11 is the CT image three-dimensional gray value and Figure 12 shows the segmentation results of different networks.

As can be seen from Figure 12, segmentation performances are improved by spatial attention mechanism, channel attention mechanism, and multiscale feature aggregation block. SAPU-Net, CAPU-Net, and MFPU-Net are superior to PU-Net in the lung cancer segmentation with complex shapes. As can be seen from the second and fourth row of the Figure 12, the there are some under-segmented phenomenon in PU-Net network, and the segmentation accuracy of APU-Net for the complex shape lesions is better than the network with a single attention mechanism. As can be seen from Table 4, comparing with those of the benchmark network PU-Net, the DSC, Recall, VOE, and RVD coefficients of SAPU-Net, CAPU-Net, and MFPU-Net are improved. Compared with spatial and channel attention mechanism, the evaluation indexes of MFPU-Net are the highest among the three mechanisms, these are 95.81%, 96.92%, 2.9%, and 2.94%, respectively, and because the multiscale feature aggregation block is to aggregate the feature maps of decoder_A and decoder_B, MFPU-Net automatically learns the image-specific weight of different scales. In conclusion, this experiment shows that the hybrid attention module and multiscale feature aggregation block used in the network are effective in improving the segmentation performance of the lung tumor.

#### 3.2.3. Comparison with Other Networks

In order to the effectiveness of the APU-Net, we compared it with SegNet [21], Wnet [22], and Attention Unet [23]. The encoder network in SegNet [21] is the convolution layer of VGG-16, decoder network is to map the low resolution encoder feature maps to full input resolution feature maps for pixel-wise classification, and the pooling indices are used to compute nonlinear upsampling in decoder. Wnet [22] is that two cascade U-Net networks are used for the segmentation of systemic bone lesions in PET/CT images of myeloma. The first U-Net network has 5 layers, and CT images are the input, while the second U-Net network has 3 layers, and the segmentation results which are the first U-Net and PET images acted as input of the second U-Net network. Attention Unet [23] is used to segment pancreatic CT images lesions, it is an unembedded attention gates in the skip connection, the size and shape of the segmentation target are automatically learned through a self-attention gate, and feature maps in encoder path and decode path are input into self-attention gate.  Figure 13 is CT image three-dimensional gray value, the segmentation results of APU-Net and other models are shown in Figure 14, and the evaluation indexes of segmentation result are shown in Table 5.

As can be seen from Table 5, the DSC, Recall, VOE, and RVD coefficients of SegNet [21] are 94.82%, 95.11%, 1.81%, and 2.04%, respectively. SegNet only uses CT single-mode images for the lesion segmentation, and the segmentation effect is not good for lesions adhered to normal tissues. As can be seen from Figure [14], there are some under-segmentation in SegNet, such as the 1^st^ row and e^th^ column, there are some oversegmentation, such as last row and e^th^ column, there are some tissue adhesions. DSC, Recall, VOE and RVD coefficients of Wnet [22] are 94.73%, 95.98%, 2.08%, and 2.17%, respectively, and its most coefficients are better than SegNet [21], such as Recall, VOE, and RVD coefficients. Final output feature maps of the first network are input into the second network by this Wnet, by making full use of the details of CT images which helps locate systemic bone lesions and PET images which can provide the metabolic information of systemic bone lesions. However, since the second network of Wnet is very shallow, and medical image feature information cannot be extract well, and lesions' edge is fuzzy in PET images, segmentation result is not good of Wnet comparing with attention mechanism. In the 2^nd^ row and f^th^ column in Figure 14, there are some under-segmentation in Wnet.

For lesions with complex shapes in the 3^rd^ and 7^th^ rows, the Wnet segmentation results are not good. As Attention Unet [23] automatically focuses on the lesion by attention gates in the skip connection, the segmentation effect is better than SegNet [21] and Wnet [22]. However, there is no metabolic information provided by PET images for lesions with complex shapes, such as the 6^th^ row and a^th^ column, and lesions adhered to normal tissues, such as the last row and a^th^ column.

## 4. Discussion

It is well known that, for patients with lung cancer, delineation of lung lesions plays an important role in the customization of treatment plan and recovery of prognosis [24]. In this study, we proposed an attention mechanism parallel U-Net which enables accurate segmentation for lung cancer. We make full use of multimodal medical images to complement lesion features and use CT images to provide anatomical information of lesions and PET images to provide functional information of lesions. We use the radar chart to show the various segmentation result indicators of each experiment. The radar chart can clearly show the various comparison result indicators of different networks.  Figure 15 is the radar chart of the segmentation index of the basic network architecture. From the chart, it can be seen that PU-Net's DSC, Recall, VOE, and RVD coefficients are all higher than U-Net and MEU-Net, and the parallel network architecture can extract more features than U-Net.

Figure 16 is a radar chart of the segmentation index of each attention mechanism network. It can be seen from the figure that except for APU-Net, the coefficients of MFPU-Net are higher than other networks. DSC and Recall coefficients increased from 95.48% to 95.91% and 95.81% to 96.92%, and VOE and RVD coefficients increased from 2.72% to 2.9% and 2.81% to 2.94%. The parallel networks with the attention mechanism are all higher than the benchmark PU-Net, so it can be concluded that the attention mechanism is effective and improves the segmentation performance of the network.

Figure 17 is a radar chart of different model segmentation indicators, and we compared SegNet, Wnet, Attention Unet, and APU-Net, respectively. The DSC, Recall, VOE, and RVD coefficients of Attention Unet [23] are 95.69%, 96.17%, 2.64%, and 2.73%, respectively. Compared with Wnet, the DSC and Recall coefficients are increased by 0.96% and 0.19%, and VOE and RVD coefficients are increased by 0.56%, respectively. It can be seen from the Figure 14 that the evaluation index coefficients of APU-Net are superior to other networks. PET, CT, and PET/CT multimodal medical image features are not used in the networks of SegNet [21] and Attention Unet [23], and single-modal medical images are only used, ignoring the complementary advantages of multimodal medical images. It is feasible to improve the segmentation performance by using multimodal medical images, and the DSC and Recall coefficients of APU-Net are increased by 0.46% and 0.26%, respectively, and VOE and RVD coefficients are increased by 0.18% and 0.23%, respectively. It is very necessary to use a parallel network to learn the features of medical images. In addition, the hybrid attention mechanism selects important feature maps and focuses on the lesions in the feature maps, which can improve the performance of network segmentation and provide a more accurate medical images segmentation, and the segmentation results are closer to the ground truth.

The paper explored two network architectures for extracting complementary information from multimodal medical images to lung tumor. The network based on multiencoder U-Net and the network based on parallel U-Net. After the adjusting parameters of the two networks, the segmentation performance shows that the based on the parallel network is superior to the network based on the three encoders. It is guessed that the parallel U-Net network has more semantic features on the decoding path than the three-encoder network, and the network has a certain impact on the performance of segmentation. Therefore, the model for extracting multimodal medical image information needs further exploration.

Due to the noninvasive characteristics of medical imaging equipment, it has become a tool for doctors to diagnose diseases [25, 26]. At present, medical image data is increasing explosively, due to their own ethical issues, medical images are difficult to obtain, and the parameters of different hospital imaging equipment are different, resulting in inconsistent medical images obtained [27]. The abovementioned problems lead to certain difficulties in feature extraction of many medical images. Therefore, the standardization of medical image data is one of the important development directions in the future.

In the future, the paper will further expand the dataset and extend the model to the segmentation of 3D lung tumors. The paper will further standardize the prescanning and scanning procedures of ^18^F-FDG PET/CT and optimize the postprocessing of data reconstruction, in order to maximize the clinical application of ^18^F-FDG PET/CT in lung malignant tumors.

## Figures and Tables

**Figure 1:** (a) Lung CT image. (b) Lung PET/CT image.

**Figure 2:** APU-Net network.

**Figure 3:** UNet_A network.

**Figure 4:** UNet_B network.

**Figure 5:** Two-modality medical image feature extraction block.

**Figure 6:** Spatial attention mechanism.

**Figure 7:** Channel attention mechanism.

**Figure 8:** Multiscale feature aggregation block.

**Figure 9:** CT image three-dimensional gray value.

**Figure 10:** Network segmentation results. (a) CT image. (b) PET/CT image. (c) and (d) PET image. (d) Ground truth. (e) U-Net segmentation result. (f) MEU-Net segmentation result of the three encoders. (g) PU-Net segmentation result.

**Figure 11:** CT image three-dimensional gray value.

**Figure 12:** Segmentation results. (a) CT image. (b) PET/CT image. (c) PET image. (d) Ground truth. (e) PU-Net segmentation result. (f) SAPU-Net segmentation result. (g) CAPU-Net segmentation result. (h) MFPU-Net segmentation result. (i) APU-Net segmentation result.

**Figure 13:** CT image three-dimensional gray value.

**Figure 14:** Comparison of segmentation results of different algorithms (a) CT image. (b) PET/CT image. (c) PET image. (d) Ground truth. (e) Segmentation results of SegNet [21]. (f) Segmentation results of Wnet [22]. (g) Segmentation results of Attention Unet [23]. (h) APU-Net segmentation results.

**Figure 15:** Radar chart of evaluation index of segmentation result.

**Figure 16:** Radar chart of segmentation index.

**Figure 17:** Radar diagram of segmentation index.

**Table 1:** Network parameters of UNet_A.

Encoder path	Feature size	Kernel size	Decoder path	Feature size	Kernel size
Block1	50 × 50	[3 × 3, 16] × 2	U1	50 × 50	[3 × 3, 16] × 2
Block2	25 × 25	[3 × 3, 32] × 2	U2	25 × 25	[3 × 3, 32] × 2
Block3	12 × 12	[3 × 3, 64] × 2	U3	12 × 12	[3 × 3, 64] × 2
Block4	6 × 6	[3 × 3,128] × 2	U4	6 × 6	[3 × 3,128] × 2
Block5	3 × 3	[3 × 3,256] × 2			

**Table 2:** Network parameters of UNet_B.

Encoder path	Feature size	Kernel size	Decoder path	Feature size	Kernel size
Block1	50 × 50	[3 × 3, 32] × 2	U1	50 × 50	[3 × 3, 32] × 2
Block2	25 × 25	[3 × 3, 64] × 2	U2	25 × 25	[3 × 3, 64] × 2
Block3	12 × 12	[3 × 3,128] × 2	U3	12 × 12	[3 × 3,128] × 2
Block4	6 × 6	[3 × 3,256] × 2	U4	6 × 6	[3 × 3,256] × 2
Block5	3 × 3	[3 × 3,512] × 2			

**Table 3:** Model segmentation index results.

Model	DSC (%)	Recall (%)	VOE (%)	RVD (%)
U-Net	95.16	94.99	2.53	2.74
MEU-Net	95.20	95.13	2.59	2.76
PU-Net	95.48	95.91	2.72	2.81

**Table 4:** Segmentation index results.

Model	DSC (%)	Recall (%)	VOE (%)	RVD (%)
PU-Net	95.48	95.91	2.72	2.81
SAPU-Net	95.79	96.35	2.87	2.9
CAPU-Net	95.78	96.47	2.88	2.89
MFPU-Net	95.81	96.92	2.9	2.94
APU-Net	96.86	97.53	3.18	3.29

**Table 5:** Comparison results between APU-Net and other networks.

Model	DSC (%)	Recall (%)	VOE (%)	RVD (%)
SegNet [21]	94.82	95.11	1.81	2.04
Wnet [22]	94.73	95.98	2.08	2.17
Attention Unet [23]	95.69	96.17	2.64	2.73
APU-Net	96.86	97.53	3.18	3.29

## Data Availability

The data used to support the findings of this study are available from the corresponding author upon request.

## References

[1] Bao S. M., Hu Q. H., Yang W. T., Wang Y., Tong Y. P., Bao W. D. (2019). Targeting epidermal growth factor receptor in non-small-cell-lung cancer: current state and future perspective. *Anti-Cancer Agents in Medicinal Chemistry (Formerly Current Medicinal Chemistry-Anti-Cancer Agents)*.

[2] Nguyen C. T. T., Petrelli F., Scuri S., Nguyen B. T., Grappasonni I. (2019). A systematic review of pharmacoeconomic evaluations of erlotinib in the first-line treatment of advanced non-small cell lung cancer. *The European Journal of Health Economics*.

[3] Astaraki M., Zakko Y., Toma Dasu I., Smedby Ö., Wang C. (2021). Benign-malignant pulmonary nodule classification in low-dose CT with convolutional features. *Physica Medica*.

[4] Zhang J., Xia Y., Zeng H., Zhang Y. (2018). NODULe: Combining constrained multi-scale LoG filters with densely dilated 3D deep convolutional neural network for pulmonary nodule detection. *Neurocomputing*.

[5] Xie H., Yang D., Sun N., Chen Z., Zhang Y. (2019). Automated pulmonary nodule detection in CT images using deep convolutional neural networks. *Pattern Recognition*.

[6] Tong G., Li Y., Chen H., Zhang Q., Jiang H. (2018). Improved U-NET network for pulmonary nodules segmentation. *Optik*.

[7] Long J., Shelhamer E., Darrell T. Fully convolutional networks for semantic segmentation.

[8] Chen L. C., Papandreou G., Kokkinos I., Murphy K., Yuille A. L. (2018). DeepLab: semantic image segmentation with deep convolutional nets, atrous convolution, and fully connected *CRFs*. *Intelligence*.

[9] Ronneberger O., Fischer P., Brox T. U-net: convolutional networks for biomedical image segmentation.

[10] Liu L., Cheng J., Quan Q., Wu F. X., Wang Y. P., Wang J. (2020). A survey on U-shaped networks in medical image segmentations. *Neurocomputing*.

[11] Khanna A., Londhe N. D., Gupta S., Semwal A. (2020). A deep residual U-Net convolutional neural network for automated lung segmentation in computed tomography images. *Biocybernetics and Biomedical Engineering*.

[12] Liu H., Cao H., Song E. (2019). A cascaded dual-pathway residual network for lung nodule segmentation in CT images. *Physica Medica*.

[13] Gridach M. (2021). PyDiNet: Pyramid dilated network for medical image segmentation. *Neural Networks*.

[14] Wang Z., Zou Y., Liu P. X. (2021). Hybrid dilation and attention residual U-Net for medical image segmentation. *Computers in Biology and Medicine*.

[15] Cao H., Liu H., Song E. (2020). Dual-branch residual network for lung nodule segmentation. *Applied Soft Computing*.

[16] Lee S., Negishi M., Urakubo H., Kasai H., Ishii S. (2020). Mu-net: multi-scale U-net for two-photon microscopy image denoising and restoration. *Neural Networks*.

[17] Takahiro Y., Tsukasa M. (2021). Detection and localization of manhole and joint covers in radar images by support vector machine and Hough transform. *Automation in Construction*.

[18] Ying Z., Ge L., Ren Y., Wang R., Wang W. A new image contrast enhancement algorithm using exposure fusion framework.

[19] Woo S., Park J., Lee J. Y., Kweon I. S. CBAM: convolutional block attention module.

[20] Gu R., Wang G., Song T. (2021). CA-Net: comprehensive attention convolutional neural networks for explainable medical image segmentation. *IEEE Transactions on Medical Imaging*.

[21] Badrinarayanan V., Kendall A., Cipolla R. (2017). SegNet: a deep convolutional encoder-decoder architecture for image segmentation. *IEEE Transactions on Pattern Analysis and Machine Intelligence*.

[22] Xu L., Tetteh G., Lipkova J. (2018). Automated whole-body bone lesion detection for multiple myeloma on 68Ga- pentixafor PET/CT imaging using deep learning methods. *Contrast Media & Molecular Imaging*.

[23] Oktay O., Schlemper J., Folgoc L. L. Attention u-net: learning where to look for the pancreas. https://arxiv.org/pdf/1804.03999v3.pdf.2021.8.26.

[24] Tao Z., Hui-ling L., Zaoli Y., Qiu S., Huo B., Dong Y. (2021). The ensemble deep learning model for novel COVID-19 on CT images. *Applied soft computing*.

[25] Rahaman M. M., Li C., Yao Y. (2020). Identification of COVID-19 samples from chest X-Ray images using deep learning: a comparison of transfer learning approaches. *Journal of X-Ray Science and Technology*.

[26] Tao Z., Huiling L., Wenwen W., Xia Y. (2019). GA-SVM based feature selection and parameter optimization in hospitalization expense. *Applied Soft Computing*.

[27] Li Y., Li C., Li X. (2022). A comprehensive review of Markov random field and conditional random field approaches in pathology image analysis. *Archives of Computational Methods in Engineering*.

